# Analysis of the Smart Medical Service Model in Super-Aged Society-UR Agency as an Example

**DOI:** 10.1155/2022/8368057

**Published:** 2022-02-28

**Authors:** Lei Zhang, Xueqing Hu

**Affiliations:** ^1^School of Urban Planning and Design, Peking University Shenzhen Graduate School, Shenzhen 518055, China; ^2^Shenzhen Talents Housing Group Co. Ltd., Shenzhen 518000, China; ^3^Xiamen Rail Transit Group Co. Ltd., Operation Branch, No. 166 Jixing Sea Wall Road, Jimei District, Xiamen, China

## Abstract

Urban Renaissance (UR) Agency in Japan is one of the world's largest public housing institutions. When faced with the serious aging problems in Japan, the Japanese implemented innovative reform, with the smart medical and pension service launched according to the characteristics of resident population and their variation trends. As it well mastered the actual needs of residents by establishing the intelligent medical system, the occupancy rate was increased. Meanwhile, the problem of inadequate local medical resources was solved, with the satisfaction of residents as well as the cultural exchange and integration within communities ameliorated, which hence realized the sustainable development of communities. In this study, the smart medical experience of Urban Renaissance Agency in Japan was explored in the hope of providing enlightenment for the development of smart communities in China. Relevant Chinese enterprises can draw lessons from the experience of community services in Japan, and via the cooperation among industries, governments, and universities, they can collaborate with universities, scientific research institutions, high-tech enterprises, district governments, and grassroots communities to give full play to the advantages of the platform and improve service quality.

## 1. Background Analysis of “Super Aging” in Japan

Japan is one of the countries most affected by aging in the world. According to the demographic statistics report released by the Ministry of Internal Affairs of Japan in 2019, the elderly population there had reached 35 million, with an aging rate as high as 28.4% [1]. According to the calculation of the Cabinet Office, the aging rate will exceed 32% in 2035. Therefore, a super-aged society has become the prime challenge of Japanese society, with a more obvious aging trend existing in the outer suburbs of Tokyo Megalopolis [2, 3]. In the latest World Health Report 2019 released by the World Health Organization (WHO), Japan ranked first in the medical system of all countries in the world [4]. However, with the development of a super-aging society, in the face of the huge financial burden of medical treatment and old-age care, Japanese governments are obliged to consider whether the existing medical and pension model is sustainable and whether a novel model is correct in this regard is required [5].

With the development of a super-aging society, the single elderly population without spouses or children is increasing annually, which brings serious challenges in terms of pensions [6]. In Japan, the serious shortage of public service resources such as pension institutions and hospitals is becoming prominent, which has become the primary challenge for the sustainable development of Japanese society [7, 8]. From the perspective of Tokyo Megalopolis, during the period from 2015 to 2025, there will be an increase of 1.75 million local elderly population [9]. Therefore, the aging of Japan, led by Tokyo, will induce a serious shortage of related resources, such as medical and old-age care resources, as given in Table 1.

Traditional medical treatment and elderly care are usually achieved by hospitalization and nursing home. However, due to practical problems such as insufficient resources, the medical industry in Japan is striving to penetrate into communities, which has progressively realized in-community medical treatment and in-community elderly care. According to the forecasting data of related institutions, the areas with a super-aging index approximate to Tokyo Megalopolis are basically consistent with the residential communities (groups) of UR Agency in Japan (Figure 1), and the demand for residential services of the main groups in UR Agency is obviously changing with the constant increase of the single and aging rates.

## 2. Changes of Rental Market in Japan and Innovation of UR Rental Housing

Based on the survey data of Mizuho Bank, by 2030, the size of Japan's housing rental market will shrink by 30% from its current size because of an aging population with fewer children. Among them, the demand for multigeneration families and young single families will be greatly reduced, whereas at the same time, the demand for elderly people, especially single elderly people, will increase greatly. Urban Renaissance (UR) Agency in Japan is one of the world's largest public housing exclusive institutions. The number of elderly people will increase from 29.24 million in 2010 to 36.85 million in 2030, while the number of people in need of care will increase from 4.91 million to 8.36 million, and the number of facilities and houses for the elderly will increase from 1.48 million to 2.5 million. Besides, the demand for a large number of age-friendly housing also stimulates government agencies and private enterprises actively to participate in the layout of age-friendly community reconstruction as well as the construction of regional medical service centers.

The full name of UR Agency is “Independent Administrative Legal Person Urban Renaissance Agency,” which controls 720,000 sets of rental homes across Japan. Since its establishment, the UR Urban Organization and its predecessors have solved the housing problems of millions of Japanese families and fulfilled the tasks during a certain historical period by providing houses for generations of families extensively. With the advent of a super-aging society, UR Agency has been endowed with new historical significance. Most of the rental houses of UR Agency are located in the suburbs where the super-aged population gathers. Especially, about 430,000 large group houses were constructed and supplied during the period from 1960 to 1970, which were difficult to meet the living needs of the existing residents in terms of area, pattern, and supporting facilities. Therefore, renovating communities to meet the living needs of the elderly has become the primary task for the UR Agency.

Moreover, with the persistent elevation of living requirements and quality of life, the all-around environmental quality along with medical and old-age care services of residential communities are important factors for improving residents' satisfaction and happiness. Based on the existing large number of public housing, the variations of market demand, regional activation, and harmonious development of communities, UR Agency correspondingly adjusts and alters its housing products, aiming to adapt to the overall requirements of the super-aged society in Japan and improve the overall quality of communities.

## 3. Reform of UR Agency and Launch of New Undertakings

To adapt to the variations of Japan's super-aged society in the future, UR Agency sets up a special committee and organized Japanese experts and scholars to perform a special study in this regard and hence formulated three future-oriented reform policies according to the reality of UR and the development tendency of Japanese society.

### 3.1. Promotion of Regional Medical Treatment and Popularization of Community Smart Medical Treatment and Welfare Facilities

Sustainable and secure family medical and nursing services are provided for the residents in UR community. For the areas with insufficient medical and nursing resources, medical institutions and elderly care facilities are attracted by means of investment promotion. To provide medical and elderly care services on a larger scale, the cooperation with public and private institutions near the community is encouraged.

### 3.2. Transformation of Smart Medical Environment and Facilities for Diverse Generations

Based on the analysis of the existing living conditions and community reality, the redesign and overall transformation should be implemented by taking safe, high-quality, and sustainable public housing as the target.

### 3.3. Creation of a Smart Information Exchange Platform: To Promote Communication among the Elderly in the Community

It provides a community platform for young groups, family groups, and elderly groups to communicate and help each other and collects opinions and suggestions from different groups as far as possible, aiming to safeguard the common interests of all stakeholders in the community and promote the harmonious community development.

## 4. Cooperation between Industries, Governments, and Education in Japan's Smart Medical Treatment: Siji-Tai District, Kashiba City, Chiba-Ken

Founded in the 1960s, Chiba-ken is not only a large-scale construction site near the JR railway station in Japan but also a typical suburb super-aging community in Japan. In recent years, as the University of Tokyo has established a new campus there, relevant scholars of the university have begun to investigate this place and put forward the idea of solving local practical problems through the cooperation between industries, governments, and the university. Under the joint efforts of the University of Tokyo, UR Agency, and local municipal governments, a new industry-government-university association, “Kashiwa Regional Super-Aged Society Comprehensive Research Association,” has been established. Aiming at the characteristics of fewer children and aging in the local areas, a series of targeted smart medical reform plans have been launched.

### 4.1. Establishment of Regional Medical Cooperation Centers to Alleviate Shortage of Medical Resources

Due to its long distance from major hospitals in Tokyo, inconvenient travel for elderly residents, and difficulties in medical treatment, UR Agency has newly established and introduced smart medical institutions here to establish a “Medical Cooperation Center,” whose main functions are as follows: first of all, after leaving from medical institutions in Tokyo, patients can continue their medical treatment at home through the Internet and Internet of things devices, the corresponding attending physicians will be recommended to the patients, and corresponding medical institutions and specialized hospitals in the area will be arranged according to the patient's situation [10]. Second, when there are insufficient medical resources, data matching can be used to provide temporary beds for patients in need of short-term hospitalization, and then, attending doctors are contracted to provide remote information support. Third, it serves as an introduction and intermediary platform for nursing, welfare services, and family nurses. Aiming at the characteristics of fewer children and aging in the local areas, a series of targeted smart medical reform plans have been launched. Fourth, it provides telemedicine consultation, medical knowledge popularization, and publicity for community residents. In addition to the above functions, the agency also cooperates with a series of groups and organizations such as the local medical doctor association and people's livelihood committee to build a 7*∗*24 hours regional medical support network through smart medical treatment to serve local communities.

### 4.2. Popularization of Home Services in Diversified Communities and Expansion of New Life Modes

To meet the demand for medical services in a super-aged society, UR provides exclusive and personalized services for the elderly in the local community by cooperating with local private enterprises [11]. In UR, for example, a “multifunctional home service center with 24-hour medical services” was established. As the center provides services for both UR residents and the residents of surrounding communities, this new service mode will be gradually popularized in the whole area [12]. The cooperation between enterprises and related organizations can bring certain benefits, and at the same time, the new pension mode is also an excellent way for promotion and popularization, which can not only improve the well-being and sense of gain of local people but also facilitate the harmonious development of the community.

## 5. Discussion

The plan of regional comprehensive smart medical centers has been implemented in more than 100 UR agencies, which enriched the local medical resources, improved the satisfaction of local and surrounding residents, and exerted a favorable impact on promoting the sustainable development of communities [13]. Meanwhile, as it well caters to the specific needs of consumers, the benefits of rental housing have been uplifted, with the medical service business also yielding certain revenues and profits. More importantly, a series of measures can be employed to better serve the community and summarize the formation and implementation processes into a set of solutions for community services, so as to provide experience templates for elderly care communities in more regions of Japan, and by extension, China [14]. Taken together, such a model is worth learning.

Relevant Chinese enterprises can draw lessons from the experience of community services in Japan, and via the cooperation among industries, governments, and universities, they can collaborate with universities, scientific research institutions, district governments, high-tech enterprises, and grassroots communities to give full play to the advantages of the platform, improve service quality, precisely analyze the resident group, and excavate residents' specific needs, so that personalized value-added services can be provided and all-round solutions can be formed. Therefore, it can be promoted in public housing communities in China. In addition to meeting the residents' needs and improving their sense of satisfaction and happiness, it can also yield value-added service benefits for enterprises while achieving certain social benefits and fulfilling corporate social responsibilities to establish favorable social images [15].

## Figures and Tables

**Figure 1:** Super-aging index of Tokyo Megalopolis (1990–2065) (Statistical Handbook of Japan 2021).

**Table 1:** Trends of ultra-aging population over 75 years old in Tokyo Megalopolis (2015–2025).

Area	Population over 75 years old		Increased number	Increasing rate
	(Ten thousand)	(Ten thousand)		
Tokyo metropolis	147.3	197.7	50.5	34.3%
Kanagawa prefecture	101.6	148.5	47.0	46.2%
Saitama prefecture	76.5	117.7	41.2	53.9%
Chiba-ken	71.7	108.2	36.6	51.0
Whole country	1645.8	2178.6	532.7	32.4

Source: Report of the Japan Conference on Entrepreneurship, the National Institute of Population Studies for Social Security 2019.

## Data Availability

The datasets used and/or analyzed during the current study are available from the corresponding author upon request.
